# NF-κB activation by *Helicobacter pylori *requires Akt-mediated phosphorylation of p65

This article has been retracted.

**DOI:** 10.1186/1471-2180-9-36

**Published:** 2009-02-12

**Authors:** Eriko Takeshima, Koh Tomimori, Hirochika Kawakami, Chie Ishikawa, Shigeki Sawada, Mariko Tomita, Masachika Senba, Fukunori Kinjo, Hitomi Mimuro, Chihiro Sasakawa, Jiro Fujita, Naoki Mori

**Affiliations:** 1 Division of Molecular Virology and Oncology, Graduate School of Medicine, University of the Ryukyus, 207 Uehara, Nishihara, Okinawa 903-0215, Japan; 2 Division of Control and Prevention of Infectious Diseases, Graduate School of Medicine, University of the Ryukyus, 207 Uehara, Nishihara, Okinawa 903-0215, Japan; 3 Division of Child Health and Welfare, Faculty of Medicine, University of the Ryukyus, 207 Uehara, Nishihara, Okinawa 903-0215, Japan; 4 The Japanese Society for the Promotion of Science (JSPS), Japan; 5 Division of Oral and Maxillofacial Functional Rehabilitation, Faculty of Medicine, University of the Ryukyus, 207 Uehara, Nishihara, Okinawa 903-0215, Japan; 6 Department of Pathology, Institute of Tropical Medicine, Nagasaki University, 1-12-4 Sakamoto, Nagasaki 852-8523, Japan; 7 Department of Endoscopy, University Hospital, University of the Ryukyus, 207 Uehara, Nishihara, Okinawa 903-0215, Japan; 8 Department of Microbiology and Immunology, Institute of Medical Science, The University of Tokyo, 4-6-1 Shirokanedai, Minato-ku, Tokyo 108-8639, Japan

## Abstract

**Background:**

The inflammatory response in *Helicobacter pylori*-infected gastric tissue is mediated by *cag *pathogenicity island (PAI)-dependent activation of nuclear factor-κB (NF-κB). Phosphatidylinositol 3-kinase (PI3K)/Akt signaling is known to play a role in NF-κB activation, but little information is available on the relationship between *H. pylori *and PI3K/Akt signaling in gastric epithelial cells. We examined whether *H. pylori *activates Akt in gastric epithelial cells, the role of *cag *PAI in this process and the role of Akt in regulating *H. pylori*-induced NF-κB activation.

**Results:**

Phosphorylated Akt was detected in epithelial cells of *H. pylori*-positive gastric tissues. Although Akt was activated in MKN45 and AGS cells by coculture with *cag *PAI-positive *H. pylori *strains, a *cag *PAI-negative mutant showed no activation of Akt. *H. pylori *also induced p65 phosphorylation. PI3K inhibitor suppressed *H. pylori*-induced p65 phosphorylation and NF-κB transactivation, as well as interleukin-8 expression. Furthermore, transfection with a dominant-negative Akt inhibited *H. pylori*-induced NF-κB transactivation. Transfection with small interference RNAs for p65 and Akt also inhibited *H. pylori*-induced interleukin-8 expression.

**Conclusion:**

The results suggest that *cag *PAI-positive *H. pylori *activates Akt in gastric epithelial cells and this may contribute to *H. pylori*-mediated NF-κB activation associated with mucosal inflammation and carcinogenesis.

## Background

*Helicobacter pylori *causes various human gastric diseases. In 10 to 20% of infected individuals, *H. pylori*-induced chronic gastric inflammation progresses to gastroduodenal ulcers, gastric cancer or gastric mucosa-associated lymphoid tissue lymphoma [1,2]. Bacterial, environmental and host genetic factors may affect the progress and outcome of gastric disease in these individuals. Virulence of individual *H. pylori *strains is one such factor responsible for severe disease, and several virulence factors have been described such as the presence of a *cag *pathogenicity island (PAI) and vacuolating cytotoxin (VacA) [3-6]. The presence of *cag *PAI genes correlates strongly with the development of ulcer diseases and gastric cancer [7-9].

Nuclear factor-κB (NF-κB) is a crucial regulator of many cellular processes, including immune response, inflammation and apoptosis [10]. It has been established that inflammation plays an important role in cancer development [11]. The five known mammalian Rel genes encode seven Rel-related proteins: RelA/p65; p105 and its processing product, p50; p100 and its processing product, p52; c-Rel; and RelB. Each contains an N-terminal Rel homology domain that mediates DNA binding, dimerization and interaction with the IκB family of NF-κB inhibitors. p65, c-Rel and RelB contain C-terminal transactivation domains, but p50 and p52 do not. The prototypical NF-κB complex is a p50–p65 heterodimer. In resting cells, NF-κB is complexed to cytoplasmic NF-κB inhibitors. IκBα is the best characterized of these inhibitors. NF-κB activation requires phosphorylation of two conserved serine residues within the N-terminal domain of IκBα (serines 32 and 36) [12]. Phosphorylation leads to ubiquitination and 26S proteasome-mediated degradation of IκBα, thereby releasing NF-κB from the complex where it translocates to the nucleus and activates various genes. Stimulation such as cytokines results in the activation of specific intracellular signaling pathways with subsequent activation of the IκB kinase (IKK) complex. This complex comprises two catalytic subunits (IKKα and IKKβ) and the regulatory subunit (IKKγ), and can phosphorylate IκBα [12]. Only *H. pylori *strains containing the *cag *PAI (*cag *PAI^+^) can direct signaling in gastric epithelial cells to activate the IKK complex and thus NF-κB, leading to the release of chemoattractants such as interleukin (IL)-8 [13]. However, the exact mechanism by which *cag *PAI^+ ^*H. pylori *strains induce activation of NF-κB in gastric epithelial cells is not clear yet. The *cag *PAI encodes a bacterial type IV secretion capable of translocating effector molecules [14]. Based on the observations that mutants of CagA, the only type IV secretion system effector protein, often induce a considerable amount of IL-8, early studies reported that CagA did not activate NF-κB or IL-8 secretion in infected cells [15,16]. However, CagA was recently reported to induce IL-8 release through NF-κB activation in time- and strain-dependent manners [17].

Protein kinases are also required for optimal NF-κB activation by targeting functional domains of NF-κB protein itself. Phosphorylation of the p65 subunit plays a key role in determining both the strength and duration of the NF-κB-mediated transcriptional response [18,19]. Sites of phosphorylation reported to date are serines 276 and 311, in the Rel-homology domain, and serines 468, 529 and 536, three phosphoacceptor sites located in the transactivation domain. Importantly, phosphorylation at serine 536 reduced the ability of p65 to bind IκBα [20] and facilitated the recruitment of TAFII31, a component of the basal transcriptional machinery [21]. Phosphorylation at serine 536 is also responsible for recruiting coactivators such as p300 [22]. The above data emphasize the importance of p65 phosphorylation at serine 536 in the function of NF-κB. In contrast, p50 phosphorylation does not regulate NF-κB activation, because p50 lacks a transactivation domain. Akt is a downstream effector of phosphatidylinositol 3-kinase (PI3K) that has been implicated in phosphorylation of serine 536 on the p65 subunit [18,19]. Akt activation also mediates multiple biological activities including increased survival, proliferation and growth of tumor cells. The present study investigated whether Akt regulates NF-κB activation in response to *H. pylori *infection.

## Results

### Immunohistochemical studies

*H. pylori*-positive gastritis biopsies of 10 patients were immunostained for phosphorylated Akt. Staining was limited to mucosal epithelial cells in all 10 patients (Figure 1A and Figure 1B), whereas no such staining was observed in the normal mucosa of all three healthy volunteers (Figure 1C and Figure 1D). Epithelial cells from three patients showed strong staining, while those of six patients showed moderate staining, and the remainder demonstrated weak staining.

**Figure 1:** **Phosphorylation of Akt in *H. pylori*-infected gastric mucosa**. Immunohistochemical detection of phosphorylated Akt in tissues of patients with *H. pylori*-positive gastritis. Serial sections of gastric biopsy specimens were stained with monoclonal antibody against phospho-Akt (serine 473). (A and B) Representative examples of mucosa from patients with *H. pylori*-positive gastritis. (C and D) Representative examples of normal mucosa. Note the positive staining for phospho-Akt in the mucosal epithelial cells of patients with *H. pylori*-positive gastritis. Original magnification, ×200.

### *Cag *PAI is required for *H. pylori*-mediated IL-8 induction in gastric epithelial cells

The *cag *PAI is a 40-kbp cluster of approximately 27 genes and encodes a type IV secretary apparatus which injects the CagA protein, and possibly other unknown proteins, into eukaryotic cells [14]. *virD4 *is one of seven genes in *cag *PAI that are virulent (*vir*) gene homologues [23]. In *H. pylori*, virD4 is thought to act as an adapter protein for the transfer of CagA protein and possibly other yet unknown proteins into the transfer channel formed by other Vir proteins in *cag *PAI [24]. The *virD4 *mutant cannot translocate CagA [24]. IL-8 cytokine is chemotactic for neutrophils and lymphocytes, and is induced in response to *H. pylori *infection. Many of the *cis*-elements that regulate IL-8 expression have been identified, including binding sites for NF-κB [25]. *H. pylori*-induced IL-8 expression is NF-κB dependent [26]. To examine the role of virulence factors in *H. pylori*-mediated NF-κB activation, we compared IL-8 induction in gastric epithelial cells infected with Δ*cag *PAI, ΔVacA, Δ*virD4 *or wild-type *H. pylori *strain. Infection with wild-type strain 26695 induced IL-8 mRNA expression in MKN45 cells, while the isogenic mutant that lacked *cag *PAI expression did not induce IL-8 mRNA expression (Figure 2A). Wild-type *H. pylori *strain but not Δ*cag *PAI strain induced IL-8 mRNA expression in AGS cells (Figure 2B). In contrast, VacA and *virD4 *null mutants induced IL-8 mRNA expression similar to the parental strain (Figure 2A). Our study on isogenic mutants derived from the 26695 strain suggests that *H. pylori cag *PAI plays an important role in the induction of IL-8 mRNA expression.

**Figure 2:** ***cag *PAI products of *H. pylori *are required for induction of IL-8 mRNA expression**. Total RNA was extracted from MKN45 (A) or AGS cells (B) infected with the wild-type strain 26695 (WT) or isogenic mutant ΔVacA, Δ*virD4 *or Δ*cag *PAI (Δ*cag*) for the indicated times and used for RT-PCR. Lane M contains markers. Representative results of three similar experiments.

### *H. pylori *activates Akt and induces phosphorylation of the NF-κB p65 subunit in gastric epithelial cells

We next examined whether coculture of gastric epithelial MKN45 cells with *H. pylori *results in activation of Akt, using Western blot analysis. As shown in Figure 3A (rows 2 and 3), phosphorylated Akt levels increased after only 30 min of coculture and this phosphorylation persisted for 3 h. There was no significant change in total Akt protein level in *H. pylori*-infected MKN45 cells (row 1). *In vitro *Akt kinase activity also increased 30 min after the addition of *H. pylori *to MKN45 cells (Figure 3A, bottom row). Since Akt is an upstream kinase implicated in p65 phosphorylation [27], we then assessed p65 phosphorylation with an antibody specific for p65 phosphorylated on serine 536. p65 phosphorylation was induced after 1 h of stimulation with *H. pylori *(Figure 3A, row 5). *H. pylori *infection also induced phosphorylated IκBα (Figure 3A, row 7). Kinetic analysis of *H. pylori*-induced degradation and resynthesis of IκBα in MKN45 cells revealed gradual increase in IκBα levels (Figure 3A, row 6). These results indicate that *H. pylori*-induced phosphorylation of IκBα leads to proteasome-mediated degradation of IκBα, thereby releasing NF-κB from the complex followed by its translocation to the nucleus to activate genes. This signal is terminated through cytoplasmic resequestration of NF-κB, which depends on IκBα synthesis, a process requiring NF-κB transcriptional activity [12]. Similar results were obtained in AGS cells (Figure 3A).

**Figure 3:** ***H. pylori *activates Akt and induces p65 phosphorylation**. (A) MKN45 or AGS cells were infected with *H. pylori *(ATCC 49503) for the indicated times. Cells were harvested, lysed and subjected to immunoblotting with the indicated antibodies. Akt *in vitro *kinase assay was performed after immunoprecipitation of Akt, with GSK-3 fusion protein serving as the exogenous substrate for Akt. Kinase reactions were analyzed by immunoblotting with monoclonal antibody for phospho-GSK-3 (serines 21 and 9). (B) The *cag *PAI of *H. pylori *is required for induction of Akt phosphorylation. MKN45 or AGS cells were infected with either the wild-type *H. pylori *strain 26695 (WT) or its isogenic *cag *PAI-lacking mutant strain (Δ*cag*) for 1 h. Cells were harvested, lysed and subjected to immunoblotting with the indicated antibodies. Representative results of three similar experiments in each panel.

We next examined whether the observed Akt activation was specific to the *cag *PAI domain, based on the above results indicating the importance of *cag *PAI expression for IL-8 induction in gastric epithelial cells *in vitro *(Figure 2). We used a wild-type *H. pylori *strain (26695) and an isogenic *cag *PAI mutant (Δ*cag *PAI). Stimulation with the wild-type strain induced Akt phosphorylation in MKN45 and AGS cells, while the isogenic mutant that lacked the expression of *cag *PAI did not (Figure 3B). These results suggest the important role of *H. pylori cag *PAI in the phosphorylation of Akt.

### *H. pylori*-induced p65 phosphorylation is PI3K-dependent

Akt is a substrate for PI3K, and thus we investigated the role of this kinase in *H. pylori*-induced Akt activation and p65 phosphorylation. As expected, inhibition of PI3K with LY294002 inhibited *H. pylori*-induced Akt activation (Figure 4A, top row), but interestingly, also abrogated *H. pylori*-induced p65 phosphorylation (Figure 4A, row 2). Despite being mutually dependent, the nuclear translocation, DNA binding and transcriptional activity of NF-κB may rely on independent regulatory elements. We investigated the role of PI3K in each of these processes by using the LY294002 inhibitor. MKN45 cells were infected with *H. pylori *and NF-κB DNA binding was assessed by electrophoretic mobility shift assay (EMSA). As shown in Figure 4B, a complex was induced in these cells within 10 min after infection with *H. pylori*. This binding activity was reduced by the addition of either cold probe or a typical NF-κB sequence derived from the CCL20 gene but not by an oligonucleotide containing the AP-1 binding site (Figure 4C, lanes 2–4). Furthermore, an NF-κB DNA complex composed of p50 and p65 was induced in MKN45 cells within 10 min after infection with *H. pylori*, but pretreatment of MKN45 cells with LY294002 did not inhibit *H. pylori*-mediated NF-κB DNA binding activity (Figure 4B and Figure 4C).

**Figure 4:** **Involvement of PI3K in *H. pylori*-mediated Akt activation and p65 phosphorylation**. (A) MKN45 cells were pretreated for 60 min with LY294002 (20 μM) or medium alone, and infected with *H. pylori *(ATCC 49503) for the indicated times (30–180 min). Cells were harvested, lysed and subjected to immunoblotting with the indicated antibodies. Akt *in vitro *kinase assays were performed as shown in Figure 3A. (B) LY294002 had no effect on the *H. pylori*-stimulated DNA binding activity of NF-κB. MKN45 cells were pretreated for 60 min with LY294002 (20 μM) or medium alone, and infected with *H. pylori *(ATCC 49503) for the indicated times for EMSA (10–60 min). (C) *H. pylori *stimulated the formation of a p65–p50 heterodimer in MKN45 cells infected with *H. pylori *(ATCC 49503) for 60 min. The cells were lysed and the competition and supershift assays were performed with the competitor oligonucleotides and the indicated antibodies (Ab), respectively.

### *H. pylori*-stimulated NF-κB transcriptional activity is dependent on PI3K/Akt

Next, to assess whether *H. pylori*-induced PI3K activity affected NF-κB transcriptional activity, we transfected MKN45 cells with an NF-κB reporter construct (κB-LUC). In contrast to the effect of LY294002 on the DNA-binding activity of NF-κB, LY294002 pretreatment caused 65% decline in *H. pylori*-stimulated luciferase expression from κB-LUC (Figure 5A). Overexpression of the dominant-negative Akt mutant also suppressed the ability of *H. pylori *to stimulate κB-LUC in a dose-dependent manner (Figure 5B). The above findings indicate that the transcriptional activity but not the DNA binding activity of NF-κB is sensitive to inhibition of Akt and PI3K.

**Figure 5:** **NF-κB-mediated transactivation induced by *H. pylori *is inhibited by either LY294002 or transfection of a dominant-negative Akt mutant**. (A) MKN45 cells were transfected with κB-LUC and phRL-TK for 24 h. Where indicated, the cells were preincubated with LY294002 (20 μM) for 60 min prior to infection with *H. pylori *(ATCC 49503). They were infected subsequently with *H. pylori *for 24 h. Luciferase activity was assayed for each sample. Readings were normalized for each sample as expressed κB-LUC over constitutively expressed phRL-TK and plotted as -fold stimulation. (B) Dominant-negative Akt blocked *H. pylori *signaling to an NF-κB-dependent promoter. MKN45 cells were cotransfected with κB-LUC and phRL-TK, together with either a vector or a construct expressing a dominant-negative Akt (Akt K179A/T308A/S473A). The cells were infected with *H. pylori *(ATCC 49503) 24 h later. Data are mean ± SD of three independent experiments.

### PI3K inhibition or transfection with small interference RNAs for p65 and Akt suppresses *H. pylori*-induced IL-8 expression

Finally, we investigated the effect of inhibition of *H. pylori*-induced PI3K activity on IL-8 expression. Pretreatment of MKN45 cells with LY294002 reduced *H. pylori*-stimulated IL-8 mRNA expression as determined by reverse transcription-polymerase chain reaction (RT-PCR) (Figure 6A). Inhibition of PI3K also significantly decreased the amount of IL-8 secreted by MKN45 cells stimulated with *H. pylori *in a dose-dependent manner (Figure 6B).

**Figure 6:** **LY294002 inhibits *H. pylori*-induced IL-8 expression and production**. (A) MKN45 cells were preincubated with LY294002 (20 μM) for 60 min prior to infection with *H. pylori *(ATCC 49503), harvested at the indicated time points and assayed for IL-8 mRNA expression by RT-PCR. Lane M contains markers. (B) LY294002 inhibits *H. pylori*-induced IL-8 production. MKN45 cells were preincubated with the indicated concentrations of LY294002 for 60 min prior to infection with *H. pylori *(ATCC 49503). For IL-8 protein determination, supernatants were collected 24 h after infection and assessed for IL-8 production by ELISA. Data are mean ± SD of three experiments.

LY294002 is a chemical inhibitor, and thus its target specificity may be questionable. Thus, small interference RNAs (siRNAs) for p65 and Akt were used to examine the role of p65 and Akt activation in the signal transduction pathway leading to IL-8 expression by *H. pylori *infection. Each siRNA specifically inhibited the expression of p65 and Akt (Figure 7). Figure 7 also shows that *H. pylori*-induced IL-8 mRNA expression was inhibited by siRNAs for p65 and Akt, confirming that p65 and Akt are important in *H. pylori*-induced IL-8 expression.

**Figure 7:** **Transfection of siRNAs for p65 and Akt inhibits *H. pylori*-induced IL-8 expression**. MKN45 cells were transfected with siRNAs for p65 and Akt, followed by stimulation with *H. pylori *(ATCC 49503) for 6 h. The RNA was subjected to RT-PCR for IL-8 and p65 mRNAs. Lane M contains markers.

## Discussion

NF-κB activation is known to regulate various cellular responses, including apoptosis, and is required for the induction of inflammatory and tissue-repair genes [10]. As reported previously [26,28], we demonstrated that *H. pylori *modulates the NF-κB system in gastric epithelial cells by inducing IκBα phosphorylation and degradation, NF-κB DNA binding activity, and NF-κB transcriptional activity. Although this investigation was a preliminary in nature in a small number of patients, we also showed that *H. pylori *infection activated Akt in epithelial cells, both *in vivo *and *in vitro*, and that this is dependent on an intact *cag *PAI *in vitro*. Interestingly, *H. pylori *also stimulated endogenous p65 phosphorylation on serine 536. Phosphorylation of p65 at serine 536 in the transactivation domain enhances the transcriptional activity of NF-κB [19]. Although previous studies using pathogenic strains containing the *cag *PAI showed NF-κB activation and cytokine expression in gastric epithelial cells [13,28], ours is the first demonstration that *cag *PAI^+ ^*H. pylori *strains induce gene expression through p65 phosphorylation, and that *H. pylori*-induced p65 phosphorylation is PI3K/Akt-dependent.

The role of PI3K/Akt signaling cascades in the regulation of NF-κB transactivation remains controversial. The present study agrees with previous investigators in demonstrating that activation of PI3K/Akt promotes the activation of p65 [29], while some others found that inhibition of the PI3K/Akt pathway augmented p65 activation [30]. We also analyzed how *H. pylori*-stimulated PI3K activation leads to the activation of NF-κB, and identified a pathway initiated by the PI3K activation that is distinct from NF-κB DNA binding. In contrast to the lack of effect of inhibition of PI3K on NF-κB DNA binding, pretreatment of MKN45 cells with LY294002 resulted in marked inhibition of *H. pylori*-stimulated p65 phosphorylation and the ability of *H. pylori *to activate NF-κB-dependent transcription. Furthermore, a dominant-negative derivative of Akt blocked the ability of *H. pylori *to activate an NF-κB-dependent promoter. Therefore, the results established a clear role of PI3K and its downstream effector Akt in modulating the transactivation potential of p65. However, the kinases and signaling pathway responsible for *H. pylori*-induced p65 phosphorylation remain unknown. Our data demonstrated for the first time that PI3K and Akt participate in *H. pylori*-mediated NF-κB transcriptional activity. Further studies are required to define the exact signaling cascade involved in bacteria-induced p65 phosphorylation and NF-κB activity.

## Conclusion

Our data demonstrated the role of PI3K/Akt in *H. pylori*-induced NF-κB transcriptional activity and subsequent IL-8 production in gastric epithelial cells. We also demonstrated an important role of PI3K/Akt in the regulation of gastric responses to *H. pylori *infection, thereby elucidating a novel mechanism that controls both transcription and gene expression in bacterial pathogenesis.

## Methods

### Antibodies and reagents

Polyclonal antibodies to Akt, phospho-Akt (threonine 308), phospho-Akt (serine 473), p65 and phospho-p65 (serine 536), as well as monoclonal antibodies to phospho-Akt (serine 473) and phospho-IκBα (serines 32 and 36) were purchased from Cell Signaling Technology (Beverly, MA, USA). Polyclonal antibodies to IκBα and NF-κB subunits p50, p65, c-Rel, p52 and RelB were obtained from Santa Cruz Biotechnology (Santa Cruz, CA, USA). Monoclonal antibody to actin was purchased from NeoMarkers (Fremont, CA, USA). PI3K inhibitor LY294002 was obtained from Calbiochem (La Jolla, CA, USA).

### Bacterial strains

*H. pylori *ATCC 49503 (American Type Culture Collection, Rockville, MD, USA) was used. Isogenic *H. pylori *mutants lacking the *cag *PAI [31], VacA and *virD4 *were also studied together with their parental wild-type strain (26695). Isogenic null mutants derived from 26695 were constructed by insertional mutagenesis, using *aphA *(conferring kanamycin resistance). *H. pylori *strains were plated on blood agar plates and incubated at 37°C for 2 days under microaerophilic conditions. Using inoculating needles, bacteria harvested from the plates were suspended in 50 ml of brucella broth containing 5% fetal bovine serum (FBS) and then cultured in a liquid medium at 37°C for 1 day in a controlled microaerophilic environment. Bacteria were harvested from the broth culture by centrifugation and then resuspended at the concentrations indicated below in antibiotic-free medium. All procedures were approved by the appropriate institutional biosafety review committees and were conducted in compliance with biohazard guidelines.

### Cell culture

The human gastric epithelial cell lines MKN45 and AGS were maintained in RPMI 1640 containing 10% FBS and antibiotics. On the day of the experiment, cells were plated on fresh serum- and antibiotic-free medium and cocultured with *H. pylori *at a final concentration of 10^7 ^colony forming unit/ml for the times indicated below.

### Tissue samples

We examined stomach biopsy specimens from 10 patients with *H. pylori *gastritis and three histopathologically-normal stomach biopsies. We analyzed the phosphorylation status of Akt at serine 473 and the presence of *H. pylori *infection by culture, serological analysis (with anti-*H. pylori *IgG antibody), rapid urease test and histological visualization with Giemsa staining. Patients with *H. pylori *gastritis showed polymorphonuclear neutrophil infiltration in the gastric epithelium in conjunction with bacteria consistent with *H. pylori*. All subjects provided informed consent before obtaining the biopsy samples.

### RT-PCR

Total RNA was extracted with Trizol (Invitrogen, Carlsbad, CA, USA). First-strand cDNA was synthesized using an RNA PCR kit (Takara Bio, Otsu, Japan). Thereafter, cDNA was amplified using 25 cycles for IL-8, 35 cycles for p65 and Akt, and 28 cycles for β-actin. The specific primers used are listed in Table 1. The thermocycling conditions for the targets were as follows: 94°C for 30 s (for IL-8 and β-actin) or for 60 s (for p65 and Akt), 60°C for 30 s (for IL-8 and β-actin) or for 60 s (for p65), or 55°C for 60 s (for Akt) and 72°C for 90 s (for IL-8 and β-actin) or for 60 s (for p65 and Akt). The PCR products were fractionated on 2% agarose gels and visualized by ethidium bromide staining.

**Table 1:** Specific primers used in RT-PCR

Primer		Sequence	Product size (bp)
IL-8	sense	5'-ATGACTTCCAAGCTGGCCGTG-3'	302
	antisense	5'-TTATGAATTCTCAGCCCTCTTCAAAAACTTCTC-3'	
p65	sense	5'-GCGGCCAAGCTTAAGATCTGCCGAGTAAAC-3'	150
	antisense	5'-GCGTGCTCTAGAGAACACAATGGCCACTTGCCG-3'	
Akt	sense	5'-ATGAGCGACGTGGCTATTGTGAAG-3'	330
	antisense	5'-GAGGCCGTCAGCCACAGTCTGGATG-3'	
β-actin	sense	5'-GTGGGGCGCCCCAGGCACCA-3'	548
	antisense	5'-CTCCTTAATGTCACGCACGATTTC-3'	

### Plasmids

The Akt dominant-negative mutant plasmid (pCMV5-K169A, T308A, S473A-Akt) encodes lysine169 (the ATP-binding site), threonine 308 and serine 473 (the phosphorylation sites) to alanine mutations. Reporter plasmid κB-LUC is a luciferase expression plasmid controlled by five tandem repeats of the NF-κB-binding sequences of the IL-2 receptor (IL-2R) α chain gene.

### Transfection and luciferase assay

MKN45 cells were transfected with 1 μg of the appropriate reporter plasmid and 5 μg of effector plasmid using Lipofectamine (Invitrogen). After 24 h, *H. pylori *was added at a ratio of bacteria to cells of 20:1 and incubated for another 24 h. Luciferase activities were measured using the dual luciferase assay system (Promega, Madison, WI, USA) and normalized by the *renilla *luciferase activity from phRL-TK.

### Preparation of nuclear extracts and EMSA

Cell pellets were swirled to a loose suspension and treated with lysis buffer (0.2 ml, containing 10 mM HEPES, pH 7.9, 10 mM KCl, 0.1 mM EDTA, 0.1 mM EGTA, 2 mM AEBSF and 1 mM DTT) with gentle mixing at 4°C. After 10 min, NP40 was added to a final concentration of 0.8% and the solution was immediately centrifuged for 5 min at 700 rpm at 4°C. The supernatant was removed carefully and the nuclei diluted immediately by the addition of lysis buffer without NP40 (1 ml). The nuclei were then recovered by centrifugation for 5 min at 700 rpm at 4°C. Finally, the remaining pellet was suspended on ice in the following extraction buffer (20 mM HEPES, pH 7.9, 0.4 M NaCl, 1 mM EDTA, 1 mM EGTA, 1 mM DTT, 2 mM AEBSF, 33 μg/ml aprotinin, 10 μg/ml leupeptin, 10 μg/ml E-64 and 10 μg/ml pepstatin A) for 30 min to obtain the nuclear fraction. All fractions were cleared by centrifugation for 15 min at 15,000 rpm. NF-κB binding activity with the NF-κB element was examined by EMSA as described previously [32]. In brief, 5 μg of nuclear extracts were preincubated in a binding buffer containing 1 μg poly(dI-dC)·poly(dI-dC) (Amersham Biosciences, Piscataway, NJ, USA), followed by the addition of a radiolabeled oligonucleotide probe containing NF-κB element from the IL-2R α chain gene (approximately 50,000 cpm). The radiolabeled oligonucleotide was prepared by filling in the overhang with the Klenow fragment of DNA polymerase I in the presence of ^32^P-dCTP and ^32^P-dATP. These mixtures were incubated for 15 min at room temperature. The DNA protein complexes were separated on a 4% polyacrylamide gel and visualized by autoradiography. For competition experiments, the cold oligonucleotide probe or competitors were used, and supershift analysis was performed using antibodies against p50, p65, c-Rel, p52 or RelB. The probe or competitors used were prepared by annealing the sense and antisense synthetic oligonucleotides as follows: for the NF-κB element of the IL-2R α chain gene, 5'-GATCCGGCAGGGGAATCTCCCTCTC-3'; for the NF-κB element of the CCL20 gene, 5'-GATCGATCAATGGGGAAAACCCCATGTG-3'; and for the AP-1 element of the IL-8 gene, 5'-GATCGTGATGACTCAGGTT-3'. The above underlined sequences are the NF-κB and AP-1 binding sites.

### Western blot analysis

Cells were lysed in a buffer containing 62.5 mM Tris-HCl, pH 6.8, 2% sodium dodecyl sulfate, 10% glycerol, 6% 2-mercaptoethanol and 0.01% bromophenol blue. Equal amounts of protein (20 μg) were subjected to electrophoresis on sodium dodecyl sulfate-polyacrylamide gels, followed by transfer to a polyvinylidene difluoride membrane and sequential probing with the specific antibodies. The enhanced chemiluminescence kit (GE Healthcare, Buckinghamshire, UK) was used for detection. The membranes were stripped in stripping buffer for probing with a different antibody. Actin served as an internal control in the Western blot procedure.

### Akt kinase assay

A non-radioactivity-based Akt kinase assay kit was purchased from Cell Signaling Technology. After immunoprecipitation of Akt, the kinase reaction was performed using the instructions provided by the manufacturer with glycogen synthase kinase (GSK)-3 fusion protein as an exogenous substrate. The kinase reaction was analyzed by immunoblotting, using an anti-phospho-GSK-3 antibody (serines 21 and 9).

### Measurement of IL-8 production

MKN45 cells were cultured in RPMI 1640 supplemented with 10% FBS in 24-well plates. Subconfluent monolayers of cells were cocultured with *H. pylori *for 24 h. The supernatants were collected and stored at -80°C. IL-8 was measured by ELISA (BioSource, Camarillo, CA, USA).

### RNA interference

The siGENOME mixtures for p65 and Akt were obtained from Dharmacon (Chicago, IL, USA). All siRNA transfections were performed using a MicroPorator (Digital Bio, Seoul, Korea), pulsed once at 1,100 V for 20 ms. The siGENOME non-targeting siRNA served as controls.

### Immunohistochemical analysis

Serial sections were deparaffinized in xylene and dehydrated using graded ethanol solutions. For better detection, sections were pretreated with ready-to-use proteinase K (Dako, Carpentaria, CA, USA) for 10 min at 37°C. This procedure increased the number of antigenic sites available for binding by the antibody. In the next step, the tissues were placed in 3% hydrogen peroxide and absolute methanol for 5 min to reduce endogenous peroxidase activity, followed by washing in PBS. Primary antibody incubations included anti-phospho Akt (serine 473) monoclonal antibody or a control IgG. After washing with PBS, the sections were covered with EnVision plus (Dako) for 40 min at 37°C and washed in PBS. Antigenic sites bound by the antibody were identified by reacting the sections with a mixture of 0.05% 3,3'-diaminobenzidine tetrahydrochloride in 50 mM Tris-HCl buffer and 0.01% hydrogen peroxide. Sections were counterstained with methyl green.

## Authors' contributions

ET carried out the experiments and drafted the manuscript. KT and HK collected and assembled the data. CI, SS and MT contributed to the experimental concept and design and provided technical support. MS performed immunohistochemical staining. HM and CS provided bacterial strains. FK and JF participated in the discussion on the study design. NM conceived of the study, and participated in its design and coordination and helped to draft the manuscript. All authors read and approved the final manuscript.
